# Effect of black cloth ointment on hypertrophic scar formation: An investigation using integrated network pharmacology and animal assay

**DOI:** 10.1111/srt.13791

**Published:** 2024-06-19

**Authors:** Qin Guo, Jin Ji, Fang Chen, Jianxin Shi, Huaxu Liu, Changle Zhu

**Affiliations:** ^1^ Department of Dermatology Affiliated Hospital of Nanjing University of Chinese Medicine Nanjing China; ^2^ Hospital for Skin Diseases Shandong First Medical University Jinan China; ^3^ Department of Pathology Affiliated Hospital of Nanjing University of Chinese Medicine Nanjing China

**Keywords:** black cloth ointment, hypertrophic scar, network pharmacology, β‐elemene

## Abstract

**Background:**

Hypertrophic scars (HS) are a common disfiguring condition in daily clinical encounters which brings a lot of anxieties and concerns to patients, but the treatment options of HS are limited. Black cloth ointment (BCO), as a cosmetic ointment applicable to facial scars, has shown promising therapeutic effects for facial scarring. However, the molecular mechanisms underlying its therapeutic effects remain unclear.

**Material and methods:**

Network pharmacology was first applied to analyze the major active components of BCO and the related signaling pathways. Subsequently, rabbit ear scar model was successfully established to determine the pharmacological effects of BCO and its active component β‐elemene on HS. Finally, the molecular mechanism of BCO and β‐elemene was analyzed by Western blot.

**Results:**

Through the network pharmacology, it showed that β‐elemene was the main active ingredient of BCO, and it could significantly improve the pathological structure of HS and reduce collagen deposition. BCO and β‐elemene could increase the expression of ER stress‐related markers and promote the increase of apoptotic proteins in the Western blot experiment and induce the apoptosis of myofibroblasts.

**Conclusions:**

Our findings indicate that the material basis for the scar‐improving effects of the BCO is β‐elemene, and cellular apoptosis is the key mechanism through which the BCO and β‐elemene exert their effects.

## 1 INTRODUCTION

Scar formation is an essential step in normal wound healing.^1^ The hallmark of the scar is the deposition of collagen in myofibroblasts.^2^ Ideally, the final scar is characterized by mild hypopigmentation, thinness, and softness. In contrast, hypertrophic scarring (HS) is an abnormal wound healing response where the scar tissue forms excessive collagen deposition.^3^ HS can cause discomfort, impaired mobility, compromised normal function, and aesthetic concerns for patients, along with significant psychological distress.^4^ Currently, due to the complexity of its cellular and molecular mechanisms which are still not completely clear, there are no satisfactory methods in the treatment or prevention of pathological scarring.

Current research indicates that the activation and proliferation of fibroblasts in the skin play a crucial role in the process of scar formation.^5^ During the repair process, quiescent fibroblasts at the site of injury are activated and differentiate into contractile myofibroblasts, synthesizing and secreting an excessive amount of extracellular matrix (ECM), depositing in the wound to act as a scaffold for other repairing cells.^6^ During normal wound healing, myofibroblasts undergo apoptosis after re‐epithelialization. In the formation of HS, myofibroblasts continue to proliferate rather than undergo apoptosis. Studies have shown an increased expression of inflammatory factors, such as IL‐1, IL‐6, and tumor necrosis factor alpha (TNF‐α), and monocyte chemoattractant protein 1 in HS.^7^ Growth factors like TGF, fibroblast growth factor (FGF), vascular endothelial growth factor (VEGF), and insulin‐like growth factor 1 (IGF1) are also elevated, further inducing cell proliferation.^8^ These problems may contribute to the differentiation of fibroblasts and the development of HS. Better and more in‐depth studies of myofibroblast formation in HS and fibrotic diseases will facilitate the development of effective therapies and therapeutic agents.

Black cloth ointment (BCO) is a traditional Chinese medicine formulation created by the esteemed expert in traditional Chinese dermatology, Mr. Zhao Bingnan.^9^ After many years of clinical application, the curative effect is exact, side effects are less, more easily accepted by the majority of doctors and patients. In this formulation, gallnut (Wubeizi) serves as the principal medicinal ingredient with functions that include clearing lung heat, stopping bleeding, and promoting wound healing. Centipede (Wugong) acts as the ministerial medicinal ingredient, known for its properties of promoting blood circulation, alleviating pain, dispersing toxicity, and relieving itching. borneol (Bingpian) functions as an adjuvant medicinal ingredient and possesses antimicrobial, antifungal, anti‐inflammatory, and analgesic properties. This formulation is often mixed with honey and aged vinegar to prevent spoilage, enhance the luster of the ointment, and improve its adhesive properties. This results in a more viscous, uniform, and easily applicable ointment on the skin, facilitating absorption. Existing data indicate that extracts from gallnut and centipede can inhibit fibroblast proliferation and collagen synthesis. The total effective rate of this treatment for post‐burn HS reaches 95%,^10^ suggesting a broad application outlook for traditional Chinese herbal medicine in the treatment of proliferative scars.

Currently, research into the mechanisms of BCO is limited. The aim of this work was to gain a deeper understanding of the effective element and potential molecular mechanisms underlying the effectiveness of BCO. This will provide a solid foundation for future in‐depth research and offer strong scientific support for its clinical efficacy. Based on our previous research,^11^ our study employed network pharmacology to identify the active components within BCO. Subsequently, it elucidated the potential molecular mechanisms via GO and KEGG enrichment analysis. Further, the pharmacological effects and mechanisms of both BCO and its active constituents were elucidated through animal experimentation. The objective of this paper is to delineate the material basis and molecular pathways through which BCO exerts its anti‐HS effects.

## 2 MATERIALS AND METHODS

### 2.1 Screening of active ingredients and targets of BCO

The standard for oral bioavailability (OB) ≥ 30% and drug‐likeness (DL) ≥ 0.18 was applied.^12^ In the Traditional Chinese Medicine Systems Pharmacology Database and Analysis Platform (TCMSP) (https://old.tcmsp‐e.com/tcmsp.php), an effective active ingredient search was conducted for the main components of the BCO, namely, gallnut, and borneol, while effective active ingredient of centipede was collecting from the literature.^13^ The gene names corresponding to the target proteins were then retrieved from the UniProt database (https://www.uniprot.org/) and organized.^14^ Additionally, relevant Venn diagrams were constructed.

### 2.2 Protein‐protein interaction network

The collected targets were imported into the STRING database(https://cn.string‐db.org/),^15^ and the protein type was set to “Homo sapiens” (human) for the operation. The minimum interaction confidence threshold was set to “medium confidence,” while all other parameters remained at their default settings. This allowed us to obtain information about protein‐protein interactions.

### 2.3 GO and KEGG enrichment analysis

The collected targets were imported into the DAVID 6.8 database (https://david.ncifcrf.gov/), with the species set to “Homo sapiens” (Human), for Gene Ontology (GO) analysis and Kyoto Encyclopedia of Genes and Genomes (KEGG) analysis.^16^ Relevant data were filtered based on a false discovery rate (FDR) of less than 0.05 for further analysis.

### 2.4 Animal experiment

Large white rabbits were adaptively housed for one week and then randomly divided into five groups: the control group, the HS model group, BCO group, the low‐dose β‐elemene group, and the high‐dose β‐elemene group.

For the control group, no specific treatment was administered. The HS model group, BCO group, the low‐dose β‐elemene group, and the high‐dose β‐elemene group underwent HS modeling. The HS model was established as follows: After anesthetizing the rabbits with chloramine (15 mg/kg) via marginal ear vein injection, under strict aseptic conditions, six circular wounds of 1 cm^2^ were created on each ear, avoiding visible blood vessels on the ventral side of the ear. The skin, subcutaneous tissue, and cartilage membrane were removed, resulting in a total of 84 wounds. The wounds were left to heal naturally after modeling, and by day 28, the scars had begun to soften, lighten in color, and become slightly elevated compared to normal skin, indicating the successful establishment of a rabbit ear HS model.

Starting 28 days after modeling, treatment was initiated. The model group received no treatment. The BCO group applied 1 g of BCO to the scar area, changing the dressing every 3 days, for a continuous 28‐day treatment. The β‐caryophyllene group received β‐elemene at doses of 40 μM (low‐dose) and 80 μM (high‐dose) applied to the scar area, changing the dressing every 3 days, for a continuous 28‐day treatment. After the treatment period, scar tissues from the model group, BCO group, and β‐elemene group, as well as normal skin from corresponding sites of the control group, were excised for various parameter measurements. The antibodies used are listed in Table 1.

**TABLE 1:** Antibody used for Western blot.

Name	Company	Art.No.
α‐SMA	Abcam	ab5694
Collagen I	Abcam	ab138492
Fibronectin	Abcam	ab2413
TIMP2	ABclonal	A1558
MMP9	ABclonal	A0289
Bax	proteintech	60267‐1‐Ig
Bcl‐2	proteintech	60178‐1‐Ig
pro‐casepase‐3	Abcam	ab32499
cleaved‐casepase‐3	Abcam	ab32042
CHOP	ABclonal	A0221
Calnexin	ABclonal	A4846
GAPDH	Abcam	ab8245

### 2.5 H&E and Masson trichrome staining

Conventional Hematoxylin and Eosin stain as well as Masson staining were done at Shanghai Ribiology Biotechnology Co, LTD (Shanghai China). Put simply, tissue sections are obtained from all control and treatment groups and formalin‐fixed and paraffin‐embedded H&E stained sections are prepared using standard well‐published protocol. Masson trichome histochemical stains are also performed using formalin‐fixed and paraffin embedded tissue sections from both control and treatment groups.^17^

### 2.6 Western blot

Take 50 mg of tissue and add it to 500 μL of lysis buffer (RIPA lysis buffer: phosphatase inhibitor: PMSF = 100:1:1). Incubate the mixture on ice for 30 min, then centrifuge at 12,000 rpm for 3 min. Collect the supernatant, and measure the protein concentration using Nanodrop One. Calculate the loading volume based on a 40 mg protein sample. Next, add loading buffer equal to 1/4 of the protein volume, and incubate at 95°C for 15 min. After cooling, store the samples at −20°C. Electrophoresis is performed using a 10% separation gel at 100 V for 60 min. Transfer the proteins to a PVDF membrane using conditions of 350 mA for 70 min. Block the membrane with 5% milk for 2 h and then incubate with the primary antibody overnight at 4°C. After incubation with the primary antibody, incubate with the secondary antibody on a shaker for 2 h. Wash the membrane with TBST three times. Prepare the exposure solution in a 1:1 ratio and apply it to the membrane. Open the exposure machine and capture the images.

### 2.7 Data analysis

The data are presented as mean ± SD. Significance between groups was determined using the Student's t‐test with GraphPad Prism 8. *P* < 0.05 is considered statistically significant.

## 3 RESULTS

### 3.1 β‐elemene is the active ingredient of the BCO

We conducted searches in TCSMP using gallnut, centipede, and borneol as retrieval objects. The results showed that both gallnut and borneol yielded relevant results, while centipede did not yield results at the time. We obtained the active ingredients and potential targets of gallnut, borneol, and centipede through TCMSP and literature searches. After removing duplicates, a total of 75 active ingredients with potential targets were identified. Among these, there were 12 from gallnut, 26 from borneol, and 39 from centipede (Figure 1A). Venn diagram analysis revealed that the common components among gallnut, centipede, and borneol were β‐caryophyllene and β‐elemene (Figure 1B). Literature research has shown that β‐elemene with anticancer activity was identified from the volatile oil of centipedes, with a content of 18.30% in the total volatile oil, which was the highest content.^18^ Therefore, we infer that β‐elemene is the main component in centipedes. Gallnut did not share common components with centipede and borneol. Through literature research, we found that gallnut mainly contains tannins, accounting for approximately 50%–70%, with gallic acid being the primary active ingredient in gallnut, possessing strong reducing properties.^19^ Additionally, gallic acid exhibits various biological activities, including anti‐inflammatory, antioxidant, antimicrobial, and antiviral properties. Therefore, it is inferred that gallic acid plays a significant role in inhibiting the proliferation of scar fibroblasts and collagen synthesis.

**FIGURE 1:** β‐elemene is the active ingredient of the BCO. (A) Number of active ingredients available for gallnut, borneol, and centipede. (B) Venn diagram analysis of common active components of gallnut, Borneol and centipede. (C) Number of potential targets for Gallnut, Borneol, and centipede. (D‐F) Protein interaction networks of gallnut, borneol, and centipede. (G) Venn diagram analysis of common active components of gallnut, Borneol and centipede.

Next, we scientifically predicted the corresponding targets for each of the collected active ingredients using TCMSP and calibrated them through the UniProt database, resulting in a total of 88 potential targets. Among these, 18 were from gallnut, 32 from borneol, and 70 from centipede (Figure 1C). By analyzing the interaction information between the drug‐target proteins using the STRING database, we then utilized Venn diagrams to identify common targets among them, which included PTGS2, MAOB, PTGS1, and TP53 (Figure 1D‐G). It was observed that these proteins also function as central nodes in the protein‐protein interaction (PPI) network (Figure 1D‐F). Subsequently, we imported the potential targets of gallnut, borneol, and centipede obtained through the aforementioned screening into the DAVID database for GO biological process analysis and KEGG pathway enrichment analysis. The results indicated involvement in biological processes such as cell proliferation and apoptosis, with associated pathways including the apoptosis pathway and the P53 signaling pathway (Figure 2A‐D) (smaller *P*‐values indicating higher likelihood).

**FIGURE 2:** GO and KEGG pathway enrichment analysis. (A) Target biological process enrichment analysis. (B) Functional enrichment analysis of target molecules. (C) Enrichment analysis of target cellular components. (D) KEGG pathway enrichment analysis of targets.

### 3.2 BCO and β‐elemene can reduce collagen deposition in rabbit ear scars

First, we successfully established a rabbit ear scar model (Figure 3A and C). After scar formation, we applied BCO made from gallnut, centipede, and borneol, as well as β‐elemene, to the rabbit ear scars (Figure 3B and D). Compared to the model group that did not receive treatment, the scars treated with BCO showed a significant reduction and even disappearance. Furthermore, we conducted histomorphological evaluation (using both routine H&E staining and Masson's trichorme staining) on respective skin tissues from control and treated groups. In comparison to the normal group, the dermis in the model group showed significant thickening, prominent collagen fiber bundles, and a noticeable increase in cell infiltration. However, after treatment with the BCO, this situation significantly improved (Figure 3E). Similarly, β‐caryophyllene also demonstrated a positive effect in scar improvement (Figure 3E), with the higher dosage of β‐elemene showing a better improvement effect, indicating that β‐elemene was indeed one of the effective components in the compound. Additionally, Masson's staining also indicated that, in comparison to the normal group, the animal model group exhibited a significant increase in collagen deposition. However, after treatment with the BCO or β‐elemene, there was a noticeable improvement in collagen deposition (Figure 3E).

**FIGURE 3:** BCO and β‐elemene improve alleviate rabbit ear scar. (A and C) Establishment of rabbit ear scar model. (B and D) Scar condition of rabbit ears after treatment of BCO and β‐elemene. (E) H&E and Masson staining of rabbit ear scar.

To further validate the inhibitory effects of the BCO and β‐elemene on the expression of collagen proteins in scar tissue, total proteins from scar tissue were extracted for immunoblot analysis. We found that following the treatment with the BCO, the expression of collagen proteins α‐SMA, Fibronectin, and α1(I)Procollagen in scar tissue significantly decreased (Figure 4A). Additionally, the expression of tissue metalloproteinase MMP‐9, which promotes collagen fiber degradation, markedly increased, while the expression of tissue metalloproteinase inhibitor TIMP‐2, which inhibits MMP‐9 enzyme activity, significantly decreased (Figure 4B). Similarly, β‐elemene also dose‐dependently reduced the expression of collagen proteins α‐SMA, Fibronectin, and α1(I)Procollagen in scar tissue (Figure 4C). It simultaneously increased the expression of MMP‐9 and decreased TIMP‐2 expression (Figure 4D).

**FIGURE 4:** BCO and β‐elemene reduced collagen deposition of rabbit ear scar. (A‐D) Western blot is used to detected the expression of Fibronectin, α1(I)procollagen, α‐SMA, MMP‐9 and TIMP2 in rabbit ear scar (*n* = 3;^*^ *P* < 0.05, ^**^ *P* < 0.01, ^***^ *P* < 0.001).

### 3.3 BCO and β‐elemene inhibite collagen expression through apoptotic pathway

In further analysis of scar tissue, it was observed that following the treatment of BCO, the apoptotic effector molecule Caspase‐3 was significantly activated in scar tissue compared to the model group, characterized by an increase in cleaved‐caspase‐3 and a decrease in pro‐caspase‐3 (Figure 5A). Concurrently, the expression of the pro‐apoptotic protein Bax increased, while the anti‐apoptotic protein Bcl‐2 decreased, resulting in a significant elevation in the Bax/Bcl‐2 ratio (Figure 5B). This indicated that the BCO improved scarring by inducing apoptosis in myofibroblasts within scar tissue.

**FIGURE 5:** BCO and β‐elemene could induce apoptosis in rabbit ear scar. (A‐D) Western blot is used to detected the expression of Cleaved‐caspase‐3, caspase‐3, Bax and Bcl‐2 in rabbit ear scar (*n* = 3;^*^ *P* < 0.05, ^**^ *P* < 0.01, ^***^ *P* < 0.001).

Similarly, compared to the model group, the activated form of the apoptotic key protein caspase‐3, cleaved‐caspase‐3, increased in response to β‐elemene (Figure 5C). Further analysis revealed that, the expression of the pro‐apoptotic protein Bax increased, while the anti‐apoptotic protein Bcl‐2 decreased, resulting in a significant elevation in the Bax/Bcl‐2 ratio (Figure 5D), indicating that β‐elemene could also exert its effects through the apoptotic pathway.

### 3.4 BCO and β‐elemene induce apoptosis through ER stress pathway

Furthermore, we also examined the expression of apoptotic factors related to the endoplasmic reticulum stress (ERS) pathway in scar tissue. It was observed that, compared to the model group, BCO significantly activated the phosphorylation of ERK (p‐ERK) (Figure 6A) and promoted the expression of CHOP and calnexin proteins mediated by ERS (Figure 6B). Thus, based on these results, we found that the BCO could induce apoptosis in myofibroblasts through the ERS pathway, contributing to the improvement of scarring.

**FIGURE 6:** BCO and β‐elemene could induce apoptosis through ER stress pathway. (A‐D) Western blot is used to detected the expression of P‐PERK, PERK, CHOP and Calenxin in rabbit ear scars (*n* = 3;^*^ *P* < 0.05, ^**^ *P* < 0.01, ^***^ *P* < 0.001).

Similarly, in line with the results of the compound, after treatment with β‐elemene, it induced phosphorylation of ERK (Figure 6C), thereby increasing the expression of ERS pathway‐related proteins CHOP and calnexin (Figure 6D).

## 4 DISCUSSION

Based on the network pharmacology model of “compound‐components‐targets,” we can rapidly analyze the effective components in the compound and identify potential targets, which to some extent elucidate the interaction between the multi‐component and multi‐target characteristics of traditional Chinese medicine compounds.^20^ This helps us better identify effective components and target actions, thereby establishing the material basis for the compound's effectiveness. In current research, we found a total of 75 main active components in the BCO through network pharmacology analysis. Venn diagram analysis revealed that the common components between centipede and borneol were β‐caryophyllene and β‐elemene. Literature research identified β‐elemene from the volatile oil of centipedes with anticancer activity, and it accounted for 18.30% of the total volatile oil, making it the highest in content.^18^ Therefore, we infer that β‐elemene was the primary volatile component responsible for centipede's effects. Borneol has pharmacological properties such as antibacterial, antifungal, anti‐inflammatory, and analgesic effects.^21^ When combined with other drugs, it can enhance their bioavailability. Gallnut did not share common components with centipede and borneol. Studies have shown that gallnut and centipede can significantly inhibit the proliferation of scar fibroblasts and collagen synthesis. Gallnut primarily contains tannins, accounting for about 50%–70%. Gallic acid, a key active ingredient in gallnut, is derived from the condensation of one molecule of glucose and 5–8 molecules of ellagic acid. Gallic acid is known for its strong reducing properties and has various biological activities, including anti‐inflammatory, antioxidant, antimicrobial, and antiviral properties.^19^, ^22^ Therefore, gallic acid likely plays a crucial role in inhibiting the proliferation of scar fibroblasts and collagen synthesis. In summary, we deduce that the main active ingredients in the hydrocolloid dressing are β‐elemene and gallic acid, serving as the material basis for its effects. Furthermore, our GO biological function analysis indicated that processes like cell proliferation and apoptosis are closely associated with the hydrocolloid dressing, and KEGG pathway enrichment analysis demonstrated the involvement of pathways such as the apoptosis pathway and the P53 signaling pathway. These findings align highly with the potential targets we selected. Past research has indicated that in HS tissue, the imbalance between fibroblast proliferation and apoptosis is a critical factor in its occurrence and development.^23^ Successful wound healing requires strict control and maintenance of the balance between ECM synthesis and degradation, which contributes to reepithelialization. HS is characterized by ECM accumulation, subsequent tissue fibrosis, and the significant role played by various types of collagens in the formation of HS.^24^ Fibroblasts are the primary ECM‐producing cells. Therefore, regulating the proliferation and apoptosis of fibroblasts is of great significance for scar repair.

Our previous research has already demonstrated that β‐elemene treatment ultimately leads to cell cycle arrest in human skin fibroblasts, followed by inducing cell apoptosis through the activation of the p53‐dependent ERS pathway. This helps reduce collagen deposition and alleviate HS.^11^ In this study, we aim to elucidate the molecular mechanisms through animal models of how the BCO and β‐elemene improve HS. The rabbit ear HS model is currently the most commonly used animal model in scar research.^25^ In our present study, to verify the pharmacological effects of BCO, as well as the effective active ingredient, β‐elemene, which was selected through network pharmacology, we successfully established the rabbit ear HS model. We conducted preliminary investigations into the effects of the BCO and β‐elemene on scar improvement. The research revealed that the BCO has a significant capacity to improve scarring, and the treatment of β‐elemene alone also exhibits a remarkable ability to enhance scarring. This indicated that β‐elemene was one of the primary active ingredients responsible for BCO effects and holds great promise as a potential therapeutic agent for scar improvement.

Existing research indicates that an imbalance between fibroblast proliferation and apoptosis may be a major contributor to the occurrence and development of scars.^26^ During the initial stages of wound healing, skin fibroblasts proliferate and differentiate into myofibroblasts, secreting a substantial amount of ECM to promote wound closure. However, if a large number of myofibroblasts persist without undergoing apoptosis at the appropriate time during the later stages of healing, they continue to secrete ECM, resulting in excessive collagen deposition, which leads to scar formation. Therefore, inducing myofibroblast apoptosis is an effective strategy to improve scarring.^27^ Our results also suggest that apoptosis was the molecular basis for the effects of BCO and β‐elemene. We treated rabbit ear HS with the BCO and β‐elemene, and following the treatment, collected scar tissues for molecular biology‐level analysis. As anticipated, the BCO could induce myofibroblast apoptosis in scar tissue through the endoplasmic reticulum pathway, leading to alleviate of scar. Furthermore, the effective active ingredient, β‐elemene, selected from the BCO, also exerts its scar‐improving effects through this pathway, further validating the scientific and effective nature of our network pharmacology screening. Therefore, these results collectively indicated that the molecular basis for the BCO containing gallnut, centipede, and borneol in improving scars was β‐elemene, and inducing myofibroblast apoptosis is a crucial molecular mechanism.

## 5 CONCLUSION

In the current study, we first identified β‐elemene as the effective element for the therapeutic effects of BCO using network pharmacology. Subsequently, the rabbit ear HS model further clarified its therapeutic actions of BCO and β‐elemene. Further investigation revealed that both BCO and β‐elemene can alleviate collagen deposition through the endoplasmic reticulum pathway, leading to the improvement of HS.

## CONFLICT OF INTEREST STATEMENT

The authors declare no conflicts of interest.

## ETHICS APPROVAL AND CONSENT TO PARTICIPATE

The animal study was approved by the Ethics Committee of the Nanjing University of Chinese Medicinec. The IRB approval number was SCXK(Su)2021‐0011, approved date was 20 November 2021. All animal experiments were conducted in accordance with the Guide for the Care and Use of Laboratory Animal by International Committees. Every effort was made to minimize the numbers and suffering of the included animals.

## Data Availability

The data that support the findings of this study are available from the corresponding author upon reasonable request.
